# Efficacy of Buqi Huoxue Decoction Combined with Cardiac Rehabilitation Nursing after Coronary Intervention in Patients with Acute ST-Segment Elevation Myocardial Infarction and Its Influence on Prognosis

**DOI:** 10.1155/2022/4008966

**Published:** 2022-03-19

**Authors:** Haiping Du, Hui Fu, Jing Yu, Zuowang Cheng, Yanhong Zhang

**Affiliations:** ^1^Department of Cardiology (I), East Hospital, Yantaishan Hospital, Yantai 264000, China; ^2^Emergency Center, the Second Affiliated Hospital of Shandong University of Traditional Chinese Medicine, Jinan 250001, China; ^3^Cardiac Function Examination Room, Affiliated Qingdao Central Hospital, Qingdao University, Qingdao 266042, China; ^4^Department of Laboratory Medicine, Zhangqiu District People's Hospital, Jinan 250200, China; ^5^Department of Hypertension, Jinan Municipal Hospital of Traditional Chinese Medicine, Jinan 250012, China

## Abstract

**Objective:**

To investigate the efficacy of the application of Buqi Huoxue Decoction combined with cardiac rehabilitation nursing for patients with acute ST-segment elevation myocardial infarction (STEMI) after percutaneous coronary intervention (PCI) and its influence on the prognosis.

**Methods:**

120 STEMI patients undergoing PCI were randomly divided into control group, cardiac care group, traditional Chinese medicine and western medicine group (TCM + WM group), and comprehensive treatment group. The control group was treated with a conventional antiplatelet therapy. On the basis of the control group, the cardiac care group was combined with cardiac care treatment. The TCM + WM group was combined with Buqi Huoxue Decoction, and the comprehensive treatment group was combined with cardiac rehabilitation care and Buqi Huoxue Decoction. The total clinical effective rate, readmission rate, and adverse reaction rate of the four groups were measured. Moreover, the myocardial injury markers (creatine kinase isoenzyme (CK-MB), cardiac troponin I (cTnI), and *α*-Hydroxybutyrate dehydrogenase (*α*-HBDH)), vascular endothelial function indexes (endothelin (ET-1) and vascular endothelial growth factor (VEGF)), cardiac function indexes (left ventricular ejection fraction (LVEF), left ventricle shortening rate (LFS), left ventricular end diastolic diameter (LVEDd), and left ventricular end systolic diameter (LVESd)), and QOL quality of life score (appetite, spirit, sleep, fatigue, and daily life) were measured.

**Results:**

The total effective rate of comprehensive treatment group was obviously increased versus to the control group and cardiac care group. The CK-MB, cTnI, *α*-HBDH, ET-1, LVEDd, and LVESd levels and SAS and SDS scores in the four groups were decreased, and VEGF, LVEF, and FS levels and QOL quality of life scores were increased after treatment. Moreover, the comprehensive treatment group has more significant changes than the other three groups. The readmission rate in comprehensive treatment group was significantly lower than the other three groups, and the difference in the incidence of adverse reactions in the four groups was not statistically significant.

**Conclusion:**

Buqi Huoxue Decoction combined with cardiac rehabilitation after PCI has a significant clinical effect on STEMI patients with PCI postoperative treatment, which can effectively reduce myocardial injury, improve the patient's cardiac function and vascular endothelial function, and improve the patient's quality of life, which can better improve the prognosis of patients.

## 1. Introduction

Acute STEMI is a subtype of coronary atherosclerotic heart disease, which can be caused by various reasons such as reduced coronary blood flow, insufficient heart oxygen supply, abnormal myocardial energy metabolism, and other pathological conditions [1]. The patient presented with an ischemic chest pain for more than 20 minutes, accompanied by nausea and vomiting, profuse sweating, dyspnea, syncope, etc., which poses a great threat to the patient's health and quality of life. In recent years, the incidence of STEMI in my country has been on the rise, and the disability rate and fatality rate are both high, and it has received extensive attention from the medical community [2]. Emergency PCI is the main method of treatment for STEMI patients. It has the advantages of less trauma and good dredging effect, and it is the most effective method to improve microcirculation [3]. Most patients can restore myocardial blood perfusion after surgery, but related studies in recent years have pointed out that some patients may form stent thrombosis after PCI, which damages the blood vessels to a certain extent and is prone to myocardial reperfusion injury and poor microcirculatory perfusion, heart failure, re-infarction, and other adverse cardiovascular events that affect the treatment effect and prognosis [4]. After undergoing surgical treatment, more patients have recurring illnesses and more complications, which increase their psychological and economic burden and adversely affect their physical rehabilitation. Therefore, while actively carrying out drug treatment, it is also necessary to do a good job of relevant intervention work. Dual antiplatelet drugs (aspirin combined with clopidogrel) are commonly used drugs after PCI. They have anticoagulant and antiplatelet effects, but they are not effective when used alone. Traditional Chinese medicine (TCM) believes that the production of STEMI is related to the poor circulation of qi and blood. PCI will damage the body and further affect the blood supply. Therefore, it is necessary to carry out the treatment of qi, blood circulation, and collaterals [5]. Cardiac rehabilitation care is to take comprehensive measures to provide long-term rehabilitation interventions to patients with cardiovascular diseases, thereby reducing the risk of recurrence or sudden death. At present, the model of cardiac rehabilitation inside and outside the hospital has broken through more time and space limitations than conventional cardiac care. Although domestic research on cardiac rehabilitation is still in its infancy, the rehabilitation system based on the theory of TCM is becoming more and more complete.

In our hospital, the combined application and research of Buqi Huoxue Decoction and cardiac rehabilitation nursing is being carried out.

## 2. Materials and Methods

### 2.1. General Information

The clinical data of 120 STEMI patients admitted to our hospital from July 2017 to January 2020 were selected for retrospective analysis. All patients underwent PCI and were randomly divided into four groups. In the control group, there were 11 females and 19 males; aged 35–69 years old, median age 52 years old; body weight 52.8–73.3 kg, median 65.4 kg; and number of implanted stents 1–3. In the cardiac care group, there were 14 female cases, 16 male cases; age 38–70 years old, median age 54 years; body weight 51.3–74.6 kg, median 66.1 kg; and number of implanted stents 2–3. In the TCM + WM group, there were 13 females and 17 males; age 37–72 years old, median age 53 years old; body weight 51.9–74.3 kg, median 64.8 kg; and the number of implanted stents is 1 to 3. In the comprehensive treatment group, there were 11 females and 19 males; age 35–71 years old, median age 53 years old; body weight 53.6–73.4 kg, median 65.7 kg; and the number of implanted stents is 1 to 3 pieces.

Inclusion criteria: All patients were to meet the relevant diagnostic criteria for acute STEMI [6], which was confirmed by echocardiography, electrocardiogram, etc., admitted to the hospital within 12 hours of onset, have indications for emergency PCI surgery, age 20–80 years old, the medical records were completed, all were aware of this trial, and sign an informed consent form. Exclusion criteria: Patients with immune system diseases, blood system diseases, malignant tumors, electrolyte disturbances, hyperthyroidism, recent anticoagulation therapy, severe infectious diseases, severe liver and kidney damage, mental or cognitive impairment, recent surgical history, previous myocardial infarction history, variant angina without fixed stenosis of coronary arteries, and allergy to the drugs used in this study were excluded. This study meets ethical requirements and was approved by the ethics committee of the abovementioned hospital (approval no. 2018042341). There was no statistically significant difference in general data such as body weight, age, gender, and number of implanted stents among the four groups.

### 2.2. Method

The control group was given a basic antiplatelet and basic nursing treatment, the cardiac care group was given cardiac rehabilitation nursing intervention on the basis of the control group, the TCM + WM group was given the treatment of Buqi Huoxue Decoction on the basis of the control group, and the comprehensive treatment group was given cardiac rehabilitation nursing and Buqi Huoxue Decoction treatment on the basis of the control group.

### 2.3. Treatment Method

Blood pressure, blood lipids, and blood sugar were controlled. The control group was treated with clopidogrel bisulfate (Approval number: J20180029, Hangzhou Sanofi Pharmaceutical Co., Ltd., 75 mg), orally, 75 mg/time, 1 time/d and aspirin enteric-coated tablets (approval number: J20171021, Bayer Healthcare Co., Ltd., 100 mg), orally, 100 mg/time, 1 time/d, continuous treatment for 30 days. The TCM + WM group took Buqi Huoxue Decoction. Prescriptions: ginseng 5 g, jujube 6 g, ginger 6 g, licorice 6 g, donkey-hide gelatin 10 g, salvia 12 g, chuanxiong 12 g, cassia twig 18 g, and Poria cocos 18 g, 18 g of cooked astragalus, 21 g of codonopsis tablets. After decoction of the abovementioned drugs, 300 mL of concoction was left, and the drugs were taken once in the morning and evening, 1 dose/d, for a total of 30 days.

### 2.4. Nursing Methods

The control group was given postoperative traditional cardiac rehabilitation nursing intervention, including basic disease knowledge health education, rehabilitation guidance, kinetic progressive exercise intervention, modular diet plan intervention, smoking cessation and alcohol restriction, medication guidance, psychological counseling, after-hospital phone calls, or family follow-up. The cardiac care group implemented a multi-dimensional comprehensive cardiac rehabilitation nursing model intervention, and implemented cardiac rehabilitation nursing strategies from three aspects: physiological state, psychological state, and patient self-management. The specific content is as follows [7]:

① Psychological aspect: The nurse should strengthen communication with patients, with a sincere, enthusiastic attitude, and a kind language; encourage patients to express their sadness, dissatisfaction, and other negative emotions; understand the source of their negative emotions; and help them eliminate negative emotions by correcting patients' misconceptions and language encouragement. The patient's questions should be answered positively in detail, and the problem should be actively dealt with. The cause of the disease, the specific methods of PCI, and related precautions should be introduced. The language of the introduction should be easy to understand, for alleviating the patient's anxiety, depression, etc., and strive for the trust of the patient. The past experience of myocardial infarction treatment in our hospital should be explained, the successful cases of treatment should be introduced, and more motivational language should be used to help patients increase their confidence in treatment and enable them to actively cooperate with subsequent cardiac rehabilitation interventions. ②Cardiac rehabilitation: The risk factors should be evaluated and a cardiac rehabilitation program based on the patient's actual condition and psychological status was formulated. Under the supervision and guidance of the head nurse, the nurse will carry out the specific implementation. The patient's condition changes should be closely monitored during the rehabilitation exercise. If there was any abnormality, the amount of activity was reduced or the activity was stopped. After the patient's condition was stable, the last activity was repeated. At the same time, the nurse should instruct patients to eat more fruits and vegetables with high dietary fiber content, taboo greasy foods, and reduce the intake of non-digestible foods such as nuts and beans to prevent constipation. 1∼3 days after PCI: The nurse keeps the patients in absolute bed rest, assists patients in changing clothes, rubbing their bodies and eating, and perform passive activities on the limbs 2 times with a single time of 10 minutes. The environment of the intensive care unit was explained, the spiritual comfort was taken into consideration, and the disease-related knowledge, triggers, pathogenesis, prognosis, treatment methods and key points of cooperation, etc., should be explained in detail. The targeted psychological counseling should be performed, and successful cases of rehabilitation should be properly listed to build self-confidence. Days 4∼5: The patients should carry out activities on the upper body, practice deep breathing slowly, 3 min/time, 2 times/d, wash their face and eat in the sitting position, take the sitting position 3 times/d, 10∼20 min/time, while being able to watch report and listen to the radio, etc.. The nurse should explain what needs to be paid attention to during the activity, and give affirmation and encouragement. Day 6∼7: The patients can sit up freely, sit down, and have a meal by the bed, sit on a chair between meals, 10 min/time, 2 times/d. Day 8∼10: The patients should walk around the bed under supervision, 10∼15 min/time, 2 times/d, be able to meet guests, and watch a peaceful movie or TV appropriately, and the nurse should explain the risk factors of the disease to the patient and their family members, and distribute the knowledge manuals on disease prevention. Day 11∼12: Patients should carry out walking training of 30∼50 m, 20 min/time, and the nurse should explain the medical treatment methods and first aid methods of the disease. Day 13∼30: The nurse should reasonably extend the walking distance and engage the patients in outdoor activities combining with the actual situation of the patient. ③After discharge from the hospital: The team will follow up regularly to guide the patient's home rehabilitation exercise, and inform the patient to return to the hospital for follow-up immediately if there is an abnormality.

### 2.5. Observation Indicators and Evaluation of Curative Effects

1. Clinical efficacy [8]. ①Remarkable effect: normal resting electrocardiogram, nitroglycerin dosage, or improvement of angina pectoris frequency and duration> 80%; total effective rate = (marked effect + effective)/total number of cases *x* 100% ②Effective: the resting ECG ST-segment rises >0.5 mm, but does not reach the normal standard, or the main lead inverted *T* wave changes from flat to upright, and at the same time, the nitroglycerin dosage or the frequency and duration of angina pectoris are improved by 50%～80%; ③ Invalid: No improvement in ECG at rest, improvement of nitroglycerin dosage or frequency, and duration of angina pectoris <50%. (2) Markers of a myocardial injury. The levels of serum CK-MB, cTnI and *α*-HBDH in the two groups were detected before and after treatment. 5 ml of fasting peripheral venous blood was collected, and then centrifuged to extract the serum and stored it at −20°C for testing, cTnI was tested with a fully automatic immunofluorescence microplate reader (Azure Biosystems), and *α*-HBDH was tested with a fully automatic biochemical analyzer (Mindray). CK-MB was detected by an enzyme-linked immunosorbent assay test (ELISA). The kits were purchased from Nanjing Jidan Biotechnology Co., Ltd., and the operation was carried out in strict accordance with the kit instructions. (3) Vascular endothelial function indicators. Radioimmunoassay was used to detect the patient's vascular ET-1 and VEGF levels. The detection equipment and detection kits were purchased from Abcam, USA. (4) Heart function indicators. JH-970 color Doppler ultrasound diagnostic apparatus (Jiangsu Jiahua Electronic Equipment Co., Ltd.) was used to detect heart function indicators, including LVEF, LFS, LVESd, and LVEDd. (5) Quality of life [9]. The QOL score scale was used to score the patient's quality of life, which was evaluated from five aspects: appetite, spirit, sleep, fatigue, and daily life. The total score was 60 points, and the score was directly proportional to the quality of life. (6) Negative emotions [10]. The SAS and SDS was used to evaluate the mood fluctuations of the patients on the first, seventh, and 30th days of treatment. The higher the score, the greater the anxiety and depression mood swings. (7) Prognosis. Follow-up for 6 months, the telephone follow-up, outpatient review, and other forms to assess the patient's prognosis, mainly including arrhythmia in the hospital, heart failure readmission, and readmission to the hospital after myocardial infarction. (8) Adverse reactions. The occurrence of adverse reactions in patients was counted, including headache, nausea and vomiting, gastrointestinal discomfort, and rash.

### 2.6. Statistical Methods

Independent repetitions of experiments were 3 times. The data were processed by the SPSS 22.0 software (IBM, NY, USA), the count data were expressed as [*n* (%)], and the measurement data were expressed as (*x* ± *s*). The *χ*2 test was used to perform statistics, and *P* < 0.05 indicated that the difference was statistically significant.

## 3. Results

### 3.1. Clinical Efficacy Was Measured in the Four Groups

The total effective rate in control group was 66.67%, the total effective rate in cardiac care group was 73.33%, the total effective rate in TCM + WM group was 80.00%, and the total effective rate in comprehensive treatment group was 96.67%. There was a significant difference between the comprehensive treatment group and control group (*P*=0.003) and between the comprehensive treatment group and cardiac care group (*P*=0.024), as shown in Table 1.

### 3.2. Levels of Myocardial Injury Markers Were Measured in the Four Groups after Treatment

The levels of CK-MB, cTnI, and *α*-HBDH in the four groups were decreased, and the levels dropped more obviously in the comprehensive treatment group compared with the other three groups after treatment (#*P* < 0.01), as shown in Figure 1.

### 3.3. Vascular Endothelial Function Indexes Were Measured in the Four Groups after Treatment

The ET-1 levels in the four groups were decreased significantly, and the levels of VEGF were increased significantly (*P* < 0.01). Moreover, the levels of the two indicators in the comprehensive treatment group changed more obviously than the other three groups (*P* < 0.01), as shown in Figure 2.

### 3.4. Cardiac Function Index Levels Were Measured in the Four Groups after Treatment

The levels of LVEF and LFS in the four groups were increased, and the comprehensive treatment group had a more significant increase in the levels of two indicators than the other three groups after treatment (#*P* < 0.01, ^*∗*^*P* < 0.05). The levels of LVEDd and LVESd in the four groups were decreased and those of the comprehensive treatment group were decreased significantly compared with the other three groups after treatment (#*P* < 0.01, ^*∗*^*P* < 0.05), as shown in Figure 3.

### 3.5. QOL Quality of Life Scores after Treatment in the Four Groups Was Compared

The scores of appetite, spirit, sleep, fatigue, and daily life of the four groups were increased and that of the comprehensive treatment group was decreased more obviously than the other three groups after treatment (*P* < 0.05), as shown in Table 2.

### 3.6. Negative Emotion Scores Were Measure in the Four Groups after Treatment

After 1 day of treatment, there was no significant difference in the scores of SAS and SDS in the four groups (*P* > 0.05). After 7 days and 30 days of treatment, the scores of both indicators in the four groups were decreased, and the scores of the comprehensive treatment group were decreased more significantly (*P* < 0.05), as shown in Figure 4.

### 3.7. Prognosis of the Four Groups Was Compared

The control group's readmission rate was 36.67%, the cardiac care group's readmission rate was 30.00%, the TCM + WM group's readmission rate was 20.00%, and the comprehensive treatment group's readmission rate was 3.33%. The comprehensive treatment group has a statistically significant difference compared with the other three groups (*P* < 0.05), as shown in Table 3.

### 3.8. Incidence of Adverse Reactions in the Four Groups Was Measured

The adverse reaction rate of the control group was 40.00%, the rate of the cardiac care group was 36.67%, the rate of the TCM + WM group was 33.33%, and the rate of the comprehensive treatment group was 30.00%. The difference between the four groups was not statistically significant (*P* > 0.05), as shown in Table 4.

## 4. Discussion

STEMI is caused by the formation of microembolisms in the blood due to abnormal blood lipid levels, leading to the formation of atherosclerotic plaques. As the disease progresses, the sclerotic plaque ruptures in the blood vessel to form thrombus and various embolic substances, block the myocardial blood vessel, affect the blood supply, and then cause myocardial ischemia [11]. In addition, overwork, low physical activity, overeating, emotional agitation, and advanced age can be used as predisposing factors, which can lead to sudden death of patients [12]. PCI surgery can perform blood perfusion to the ischemic myocardium, thereby improving the patient's myocardial ischemia, but it can also induce necrosis of myocardial tissues and cause irreversible damage. Related studies have found that although PCI can dredge blood vessels and it can also induce oxidative stress and inflammation [13]. Some patients can hardly achieve the desired results after treatment. Moreover, the use of conventional nursing methods after surgery can only control the patient's condition. The complications and quality of life cannot be effectively controlled, and the prognostic effect can be reduced. In order to reduce the damage to the myocardium, clinical treatment is often supplemented by western medicine [14], but the effect is not good.

Chinese medicine believes that STEMI is located in the heart and is also related to the kidneys, lungs, liver, spleen, and other organs [15]. PCI will damage the righteous qi, further aggravate the symptoms of qi stagnation and blood stasis, and affect the rehabilitation effect. Therefore, activating blood, replenishing qi, and dredging collaterals are the key points in the treatment. In this study, Fuling and Codonopsis have the effects of invigorating the spleen and dampness, replenishing water and qi, calming the mind, and nourishing the heart. Guizhi and *Astragalus* have the function of strengthening the body, supplement Yang Qi, and warming the meridians. Ligusticum chuanxiong and Danshen have the functions of regulating qi and dispelling stagnation, promoting blood circulation and collaterals, replenishing qi, and analgesia. Ginseng nourishes the middle energy and nourishes vital energy. Jujube invigorates the intestines and nourishes blood. Donkey-hide gelatin nourishes yin and nourishes blood. Ginger restores yang and strengthens the pulse, warms the middle, and nourishes the qi. Licorice regulates the qi and harmonizes various medicines to make medicine [16–19]. The combined use of various medicines has the effects of replenishing qi, activating blood, dredging collaterals, and relieving pain. Although exercise cardiac rehabilitation in the past cardiac rehabilitation nursing model has achieved certain results in improving the patient's vascular endothelial function, stabilizing coronary plaques, and promoting the construction of collateral circulation. However, it cannot cover all aspects of nursing care and is more limited. Therefore, this study carried out cardiac rehabilitation care based on the three dimensions of physical needs, psychology, and STEMI patient self-management [20–22]. The nursing method can improve the patient's disease cognition and compliance, so as to reduce the risk of adverse cardiac events, and play a role in alleviating the patient's anxiety and tension. It can inhibit the excitability of the sympathetic nerve of the patient, slow down the induced vasoconstriction, increase the heart rate, and increase the blood pressure. Appropriate exercise can take into account physical and mental recovery, coherent and coordinated movements, and smooth stretching, making it easier for patients to operate, master, regulate their functions, and strengthen their bodies. It is similar to the basic concept of modern cardiac rehabilitation. The resistance training given to patients in this study is for patients' exercise endurance. The effect of improving the quality of life is obvious. It not only helps relieve the patient's lumbar muscle fatigue, improves gastrointestinal motility, and facilitates blood circulation, but also reduces myocardial oxygen consumption, improves myocardial contractility, increases LVEF, and promotes heart function recovery.

In this study, the total effective rate of postoperative treatment was 96.67% in the comprehensive treatment group, which was higher than the other three groups. cTnI is a regulatory protein of myocardial muscle tissue contraction and a marker of myocardial injury and necrosis. The increase in its level indicates damage to myocardial tissues and functions [23]. CK-MB is a creatine kinase that exists on cardiomyocytes and plays an important role in the activity of cardiomyocytes [24]. In clinical practice, CK-MB, cTnI, and *α*-HBDH can reflect the degree of myocardial necrosis and are important indicators for efficacy evaluation and prognosis evaluation. In this study, these levels in the four groups were significantly reduced after treatment, and the levels in the comprehensive treatment group were significantly lower than the other three groups. The cardiac function indexes LVEF, FS, LVEDd, and LVESd of patients in the comprehensive treatment group were significantly improved compared with the other three groups. It shows that the clinical efficacy of Buqi Huoxue Decoction combined with cardiac rehabilitation nursing treatment has been significantly improved. It has the effects of inhibiting platelet aggregation, reducing blood viscosity and blood coagulation, and improving microcirculation. It can better improve the patient's cardiac function index level and achieve better prognostic effects. In STEMI patients, the vascular endothelial function is also damaged due to ischemia and hypoxia. ET-1 can reflect the degree of damage to the patient's vascular endothelial function, and its increase can promote a myocardial ischemia reperfusion injury in patients with acute myocardial infarction, and aggravate the condition [25]. The ET-1 level of patients in the comprehensive treatment group was significantly lower than the other three groups, and the VEGF level was significantly higher than the other three groups, indicating that Buqi Huoxue Decoction combined with cardiac rehabilitation care can be adjusted by improving the interstitial remodeling of myocardial cells. The tension of myocardial blood vessels increases myocardial blood supply and promotes myocardial microangiogenesis. The level of VEGF is also increased, the vascular endothelial function is improved, and myocardial blood supply and myocardial contractility are restored. The adverse reactions after the comprehensive treatment group increased TCM treatment did not increase significantly, and the readmission rate was significantly lower than the other three groups, suggesting a good safety and prognosis.

This study has certain limitations: the sample size is small, and long-term observation of selected patients has not been performed, so the impact on the long-term prognosis of patient needs to be further observed.

In summary, the treatment of STEMI patients after PCI with Buqi Huoxue Decoction combined with cardiac rehabilitation can improve the treatment effect, improve the heart function, improve the quality of life, reduce the occurrence of adverse reactions and readmission rates, and have a good prognosis of patients.

## Figures and Tables

**Figure 1:** Detection of myocardial injury markers levels in the four groups after treatment. (a) Detection of CK-MB levels after treatment. (b) Detection of cTnI levels after treatment. (c) Detection of *α*-HBDH levels after treatment. ^#^*P* < 0.05.

**Figure 2:** Detection of vascular endothelial function indexes of the four groups after treatment. (a) Detection of ET-1 levels after treatment. (b) Comparison of VEGF levels after treatment. ^*∗*^*P* < 0.01, #*P* < 0.01.

**Figure 3:** Detection of four groups of cardiac function index levels after treatment. (a) Detection of LVEF levels after treatment in the four groups. (b) Detection of LFS levels after treatment in the four groups. (c) Detection of LVEDd levels after treatment in the four groups. (d) Detection of LVESd levels after treatment in the four groups. #*P* < 0.01, ^*∗*^*P* < 0.05.

**Figure 4:** Measurement of negative emotion scores in the four groups after treatment. (a) Measurement of SAS scores after treatment for 1, 7, and 30 days. (b) Measurement of SDS scores after treatment for 1, 7, and 30 days. ^*∗*^*P* < 0.05, ^#^*P* < 0.05.

**Table 1:** Measurement of the clinical efficacy in the four groups (*n*, %).

Group	*n*	Remarkable effect	Effective	Invalid	Total effective rate (%)
Control group	30	9	11	10	20 (66.67)
Cardiac care group	30	12	10	8	22 (73.33)
TCM + WM group	30	15	9	6	24 (80.00)
Comprehensive treatment group	30	20	9	1	29 (96.67)
*X* ^*2*^_*1*_	0.698		P1	0.705	
*X* ^*2*^_*2*_	2.700		P2	0.259	
*X* ^*2*^_*3*_	11.736		P3	0.003	
*X* ^*2*^_*4*_	7.497		P4	0.024	
*X* ^*2*^_*5*_	4.286		P5	0.117	

*X* ^2^_1_, P1 indicate Cardiac care group compared with control group; *X*^2^_2_, P2 indicate TCM + WM group compared with control group; *X*^2^_3_, P3 indicate comprehensive treatment group compared with control group; *X*^2^_4_, P4 indicate cardiac care group compared with comprehensive treatment group; *X*^2^_5_, P5 indicate TCM + WM group compared with comprehensive treatment group.

**Table 2:** Detection of QOL quality of life scores after treatment in the four groups (*n* = 30, *x* ± *s*).

Group	Appetite	Spirit	Sleep	Fatigue	Daily life
Control group					
Before treatment	31.93 ± 4.93	32.43 ± 2.64	31.93 ± 4.92	31.93 ± 5.00	31.77 ± 4.88
After treatment	39.70 ± 2.54	39.80 ± 2.81	40.07 ± 2.52	40.17 ± 2.98	40.30 ± 2.84

Cardiac care group					
Before treatment	33.10 ± 4.91	33.43 ± 2.64	33.13 ± 4.87	33.47 ± 5.41	33.60 ± 5.34
After treatment	51.60 ± 2.43#	51.67 ± 2.48#	52.03 ± 2.57#	52.23 ± 5.84#	52.43 ± 2.92^#^

TCM + WM group					
Before treatment	31.83 ± 4.89	30.83 ± 2.78	32.13 ± 5.48	32.70 ± 5.67	32.73 ± 5.64
After treatment	46.43 ± 2.40#	46.47 ± 2.61#	46.53 ± 2.52#	46.57 ± 2.94#	46.57 ± 3.05^#^

Comprehensive treatment group					
Before treatment	31.63 ± 4.97	32.27 ± 2.15	31.77 ± 5.10	31.93 ± 5.65	31.87 ± 5.85
After treatment	53.87 ± 1.93*∗*^#^	53.97 ± 2.17*∗*^#^	53.93 ± 4.86*∗*^#^	53.80 ± 1.88*∗*^#^	53.80 ± 2.02*∗*^#^

^#^ *P* < 0.05 vs control group, ^*∗*^*P* < 0.05 vs other three group.

**Table 3:** Measurement of the prognosis of the four groups (*n* = 30, %).

Group	Readmission rate			Total incidence
	Arrhythmia	Heart failure	Myocardial infarction recurrence	
Control group	4	4	3	11 (36.67)
Cardiac care group	3	3	3	9 (30.00)
TCM + WM group	3	2	1	6 (20.00)
Comprehensive treatment group	0*∗*^#^	0*∗*^#^	1*∗*^#^	1 (3.33)*∗*^#^

#*P* < 0.05 vs control group, ^*∗*^*P* < 0.05 vs other three group.

**Table 4:** Detection of adverse reactions' incidence in the four groups (*n* = 30, %).

Group	Headache	Gastrointestinal discomfort	Rash	Nausea and vomiting	Total incidence
Control group	5	3	2	2	12 (40.00)
Cardiac care group	3	3	3	2	11 (36.67)
TCM + WM group	4	2	3	1	10 (33.33)
Comprehensive treatment group	2*∗*^#^	2*∗*^#^	2*∗*^#^	3*∗*^#^	9 (30.00)*∗*^#^

#*P* < 0.05 vs control group, ^*∗*^*P* < 0.05 vs other three group.

## Data Availability

The data used to support the findings of this study are available on reasonable request from the corresponding author.
